# Histone deacetylase inhibitors vorinostat and panobinostat induce G1 cell cycle arrest and apoptosis in multidrug resistant sarcoma cell lines

**DOI:** 10.18632/oncotarget.20460

**Published:** 2017-08-24

**Authors:** Eva Bernhart, Nicole Stuendl, Heike Kaltenegger, Christian Windpassinger, Nicholas Donohue, Andreas Leithner, Birgit Lohberger

**Affiliations:** ^1^ Institute of Molecular Biology and Biochemistry, Medical University of Graz, 8010 Graz, Austria; ^2^ Department of Orthopedics and Trauma, Medical University of Graz, 8036 Graz, Austria; ^3^ Institute of Human Genetics, Medical University of Graz, 8010 Graz, Austria

**Keywords:** G1 cell cycle arrest, vorinostat, belinostat, sarcoma, panobinostat

## Abstract

Synovial sarcoma and high grade chondrosarcoma are characterized by their lack of response to conventional cytotoxic chemotherapy, the tendency to develop lung metastases, and low survival rates.

Research within the field prioritizes the development and expansion of new treatment options for dealing with unresectable or metastatic diseases. Numerous clinical trials using histone deacetylases inhibitors (HDACi) have shown specific efficacy as an active antitumor agent for treating a variety of solid tumors. However, as of yet the effect of different HDACi on synovial- and chondrosarcoma cells has not been investigated. In this study, vorinostat (SAHA), panobinostat (LBH-589), and belinostat (PXD101) decreased cell viability of synovial sarcoma (SW-982) and chondrosarcoma (SW-1353) cells in a time- and dose dependent manner and arrested SW-982 cells in the G1/S phase. Western blot analysis determined the responsible cell cycle regulator proteins. In addition, we found apoptotic induction by caspase 3/7 activity, caspase 3 cleavage, and PARP cleavage. In SW-1353 cells only SAHA showed comparable effects. Noteworthy, all HDACi tested had synergistic effects with the topoisomerase II inhibitor doxorubicin in SW-1353 chondrosarcoma cells making the cells more sensitive to the chemotherapeutic drug.

Our results show for the first time that SAHA and LBH-589 reduced viability of sarcoma cells and arrested them at the G1/S checkpoint, while also inducing apoptosis and enhancing chemotherapeutic sensitivity, especially in chondrosarcoma cells. These data demonstrate the exciting potential of HDACi for use in sarcoma treatment.

## INTRODUCTION

Soft tissue sarcomas (STS) are a rare class of malignant tumors with varying histology and mostly aggressive characteristics, both locally and in the formation of distant metastases [1]. STS frequently exhibit chemotherapeutic resistance and an increased metastatic potential following unsuccessful cancer treatment. Particularly in chondrosarcoma and synovial sarcoma, the efficacy of chemotherapeutic agents is limited and development and discovery of new lead substances is urgently required [2, 3].

Synovial sarcoma is the fourth most common type of STS and has a tendency to arise in the soft tissue surrounding larger joints, and occurs predominantly in younger adults with a median age of diagnosis of 35 years [4]. Standard treatment for synovial sarcoma is tumor resection frequently accompanied by radiotherapy and/or chemotherapy, although some data suggest that therapies in addition to surgery substantially increase long-term metastatic risks [5]. While many factors that influence synovial sarcoma patient outcome have been identified, tumor behavior remains highly unpredictable [6]. Chondrosarcoma denotes a heterogeneous group of neoplasms, comprised of tumor cells that share the common characteristic of producing extracellular matrix components in cartilage tissue [7]. With an incidence of 1:50,000 chondrosarcoma typically occurs in adults in their 3^rd^ to 6^th^ decade of life and represents the second most common primary malignant bone tumor in a large epidemiologic series [8]. The balance of histone acetylation and deacetylation is an epigenetic layer with a critical role in the regulation of gene expression. Histone acetylation induced by histone acetyl transferases (HATs) is associated with gene transcription, while histone hypoacetylation induced by histone deacetylase (HDAC) activity is associated with gene silencing [9]. HDACs play an important role in epigenetic gene regulation by deacetylating both, histone and non-histone (e.g. transcription factors) proteins, thereby regulating important cellular processes such as cell-cycle progression and apoptosis [10, 11]. To date, the HDAC family is divided into 4 classes: class I, IIa/b, III/sirtuins, and IV, comprising a total of 18 enzymes. A key element that allows cancer development is the deregulation of histone acetylation as well as the mutation and/or aberrant expression of HDACs. Specifically, class I subfamily members HDAC 1, 2, 3, and 8 are deregulated in many cancer types contributing to enhanced cell cycle progression and proliferation. However, the specific roles of individual HDACs in cancer are not yet fully understood, but deciphering these specificities could potentially support development of targeted therapeutics for diverse tumor entities [12, 13]. Interestingly, inhibition of HDAC activity by small molecules has been shown to provide a therapeutic benefit to patients with diverse diseases including malignancies [14]. Although already in clinical trials [15], the molecular responsibilities for the cellular mechanisms underlying HDAC inhibitor (HDACi) induced effects on cell cycle progression and cell proliferation especially in STS remains to be clarified. Cell proliferation is a tightly controlled process consisting of multiple checkpoints which direct cell cycle progression. Transitions between G1, S, and G2/M phases are regulated by coordinated actions of cyclins, cyclin-dependent kinases (CDKs), and CDK inhibitors. All of these can be modulated by diverse intracellular signals transduced from extracellular growth cues [16].

The aim of the current study was to investigate the effects of the HDACi suberoylanilide hydroxamic acid (vorinostat, SAHA), panobinostat (LBH-589), and belinostat (PXD101) on cell viability, cell cycle distribution, expression of cell cycle regulators and apoptosis in two different multidrug resistant sarcoma cell lines. Furthermore, the effect of combined treatment with HDACi and doxorubicin, a chemotherapeutic agent frequently used in the clinical setting was analyzed.

## RESULTS

### HDAC inhibitors reduced proliferation of sarcoma cells

To investigate the influence of HDAC inhibitors on sarcoma cell growth, SW-982 (synovial sarcoma) and SW-1353 (chondrosarcoma) cells were exposed to SAHA (0.5, 1.0, 2.5, 5.0, 10.0, 15.0 μM), LBH-589 (0.01, 0.05, 0.1, 0.25, 0.5, 1.0, 5.0 μM), or PXD101 (0.5, 1.0, 2.5, 5.0 μM) for 48 h. Cell viability was determined using a MTS based assay. HDACi treatment induced dose-dependent inhibition of cell viability in both cell lines with calculated IC_50_ values of 8.6 μM, 0.1 μM, and 1.4 μM (SW-982), as well as 2.0 μM, 0.02 μM, and 2.6 μM (SW-1353) for SAHA, LBH-589, and PXD101, respectively (Figure 1). DMSO (0.5%) used as vehicle control, had no effect on cell growth (data not shown).

**Figure 1:** Effect of HDACi on sarcoma cell viability SW-982 **(A)** and SW-1353 **(B)** cells were treated with 0-15 μM vorinostat (SAHA), 0-5 μM panobinostat (LBH-589) or 0-5 μM belinostat (PXD101) for 48 h to examine dose-dependent inhibitory effects. Cell viability was determined by MTS assay. Results were normalized to vehicle controls (DMSO) and represent mean ± SD of at least three independent experiments done in quadruplicates. A four-parameter logistic model determined IC_50_ values of 8.6 μM (SAHA), 0.1 μM (LBH-589) and 1.4 μM (PXD101) for SW-982 cells, as well as 2.0 μM (SAHA), 0.02 μM (LBH-589) and 2.6 μM (PXD101) for SW-1353 cells.

### Expression of Class I HDACs in SW-982 and SW-1353 cells

After treatment with the respective IC_50_ and IC_75_ concentrations of SAHA, LBH-589, and PXD101 for 48 h, whole cell lysates were extracted from the cells and prepared for western blot analysis. In SW-982 and SW-1353 cells, all class I HDACs were equally expressed as shown by immunoblot analysis (Figure 2). Treatment with the respective IC_50_ and IC_75_ concentrations of SAHA, LBH-589, and PXD101 for 48 h had no effect on HDAC protein levels, only high concentrations of SAHA slightly reduced HDAC8 expression.

**Figure 2:** Expression of Class I HDACs in SW-982 and SW-1353 cells Protein expression of Class I HDAC members HDAC1, -2, -3, and -8 in SW-982 and SW-1353 cells was evaluated by immunoblotting under control conditions and in the presence of the IC_50_ and IC_75_ concentrations of the HDACi SAHA, LBH-589, and PXD101 for 48 h. β-actin was used as loading control. Δ, fold change normalized to controls (mean±SD of n = 3).

### Effect of HDACi on cell cycle distribution

Next, FACS analysis was performed to determine the cell cycle profiles of SW-982 and SW-1353 cells when exposed to HDAC inhibitors at their respective IC_50_ concentrations for 48 h. Untreated cells were measured as controls. Representative FACS measurements are presented in Figure 3A. The percentages of the cell cycle distribution across the population are listed in Table 1, the graphical representations of the G0/G1-, S- and G2/M-values are shown in Figure 3B. SAHA treatment caused a highly significant increase in the number of cells in G1 phase compared to controls in both SW-982 and SW-1353 cells, which was accompanied by a decrease in the number of S phase cells, indicating a G1/S phase arrest. In contrast, LBH-589 and - to a lesser extent - PXD101 caused this significant effect only in the synovial sarcoma cell line SW-982. However, both drugs showed tendency to enhance cell numbers in G0/G1 after 24 hours comparable to SAHA (control: 63%, SAHA: 68%, LBH-589: 69%, PXD101: 69%; data not shown).

**Figure 3:** Influence of HDACi on cell cycle distribution **(A)** Representative FACS cell cycle measurements after 48 h exposure to the respective IC_50_ concentrations of HDACi (8.6 μM (SAHA), 0.1 μM (LBH-589), and 1.4 μM (PXD101) for SW-982 cells; 2.0 μM (SAHA), 0.02 μM (LBH-589), and 2.6 μM (PXD101) for SW-1353 cells). Percentages of G_0_/G_1_ are given. **(B)** Graphical representations of the cell cycle distribution of SW-982 and SW-1353 under control conditions and in response to HDACi treatment (IC_50_ for 48 h). Cell populations in G0/G1, S, and G2/M phases are given as percentage of total cells (mean of n = 5; *p < 0.05). Data represent the mean values from 5 independent experiments and the detailed analysis is given in Table 1.

**Table 1:** Cell cycle distribution of sarcoma cell lines after 24 and 48 h exposure to their respective IC_50_ values of HDACi (8.6 μM (SAHA), 0.1 μM (LBH-589) and 1.4 μM (PXD101) for SW-982 cells; 2.0 μM (SAHA), 0.02 μM (LBH-589) and 2.6 μM (PXD101) for SW-1353 cells) (n = 5; mean ± SD; *p < 0.05, **p < 0.01, ***p < 0.001)

Cell line	HDACi	Time	G_0_G_1_(%)	S (%)	G2/M (%)
SW-982	*control*	24 h	*55.92±8.13*	*25.06±4.55*	*19.03±5.16*
	SAHA	24 h	81.38±8.66**	1.46±0.88**	17.15±7.81
	LBH-589	24 h	82.93±5.49**	1.24±0.91**	15.83±4.79
	PXD101	24 h	82.06±6.07**	1.51±1.13**	16.43±5.44
	*control*	48 h	*67.35±6.83*	*19.89±5.18*	*12.76±2.27*
	SAHA	48 h	87.72±3.10***	3.74±1.37***	8.45±2.23**
	LBH-589	48 h	87.67±2.70***	4.03±1.74***	8.31±3.03*
	PXD101	48 h	77.03±7.48*	12.07±5.17*	10.90±5.51
SW-1353	*control*	24 h	*63.03±4.65*	*16.73±3.77*	*20.25±0.88*
	SAHA	24 h	67.89±3.64	7.28±3.98*	24.82±6.55
	LBH-589	24 h	69.43±2.24	15.02±2.47	15.55±1.02*
	PXD101	24 h	68.72±3.57	10.14±8.18	21.14±5.73
	*control*	48 h	*55.03±9.06*	*21.42±8.81*	*23.28±2.99*
	SAHA	48 h	75.04±8.48**	2.85±1.94**	22.11±8.37
	LBH-589	48 h	56.70±10.31	19.93±3.56	23.36±6.90
	PXD101	48 h	53.08±4.77	21.91±5.54	25.01±2.31

### Effect of HDACi on cell cycle regulator proteins

To confirm cell cycle analysis data, we examined the expression and activation of cell cycle checkpoint proteins using western blot analysis (Figure 4). Consistent with the inhibition of G1-to-S phase progression we found decreased cyclin D1 expression and decreased phosphorylation of CDK4 and CDK2 in SW-982 cells in response to SAHA, LBH-589, and PXD101. Similar decreases in cyclin D1 expression and CDK4 and CDK2 phosphorylation were measured in SW-1353 cells after SAHA treatment. In SW-1353, treatment with LBH-582 and PXD101 led to diminished phosphorylation of CDK4, although only small changes in cell cycle distribution were observed. Consistent with the fact that cyclin E expression reaches a maximum during the late G1 phase, in SW-982 cells the cyclin E level increased significantly after HDACi treatment, and in SW-1353 particularly after SAHA treatment. Moreover, cyclin B1 and CDK1 expression was dormant after HDACi treatment in SW-982 cells and downregulated in SW-1353.

**Figure 4:** Influence of HDACi on cell cycle proteins regulating the G1/S transition Western blot analysis of phosphorylated and total cyclin dependent kinases (CDKs) and their modulating cyclins in response to HDACi treatment for 48 h. One representative immunoblot out of three is shown. β-actin was used as loading control. Δ, fold change normalized to controls (mean±SD of n = 3).

Since HDACi-induced G1/S phase arrest is mainly dependent on transcriptional changes in cell cycle regulatory genes [17, 18], we examined the expression of CDK inhibitors p21 and p27 (Figure 4). In SW-982 cells p21 was significantly upregulated in response to IC_50_ concentrations of SAHA, LBH-589, and PXD101. In SW-1353 cells, SAHA induced a pronounced increase in p21 expression, whereas only weak induction of p21 expression was observed after LBH-589 and PXD101 treatment. In contrast, no expression changes of p27 were detected in response to HDACi treatment. Interestingly, we found no up-regulation but a slight down-regulation of p53 in SW-982 cells expressing wild-type p53 [19], although phosphorylated histone variant H2AX, a biomarker for DNA double strand breaks (DBS), was elevated in response to all three HDAC inhibitors used (Figure 5). To verify the p53 status of SW-982 cells we performed Sanger sequencing of the coding regions of TP53 (NCBI Reference Sequence: NM 000549) revealing no pathogenic variants. Similarly, in p53-mutant SW-1353 cells a clear downregulation of p53 protein levels was observed after SAHA treatment. Phosphorylation of H2AX was most pronounced after SAHA treatment, whereas LBH-589 and PXD101 induced only weak activation.

**Figure 5:** Effect of HDACi on tumor suppressor proteins p53, p21, and p27 and on DBS marker pH2AX Analysis of tumor suppressor protein and pH2AX expression was performed by immunoblotting after 48 h treatment with HDACi SAHA, LBH-589, and PXD101. One representative blot out of three is shown. β-actin was used as loading control. Δ represents fold change normalized to controls (mean±SD of n = 3).

### Induction of apoptosis

The induction of apoptosis by HDAC inhibitors was investigated by quantitative measurement of caspase 3/7 activity using the Caspase-Glo^®^ 3/7 assay and flow cytometric analysis (FACS) of caspase-3 cleavage. In addition, proteolytic cleavage of poly (ADP ribose) polymerase (PARP) as an indicative marker of apoptosis was evaluated. Figure 6A-6C shows the different effects of HDACi in terms of apoptosis. In SW-982 cells, caspase 3/7 activity was increased in response to SAHA, PXD101, LBH-589 treatment after 24 and 48 hours (p < 0.05) up to 23%. Similarly, treatment with HDACi for 24, 48, and 72 hours induced caspase 3/7 activity in SW-1353 cells. Especially SAHA caused a prominent 3-fold activation of caspase 3/7 (Figure 6A). In addition, flow cytometry analysis revealed a significant cleavage of caspase-3 in response to SAHA treatment in both, synovial sarcoma (21%) and chondrosarcoma cells (28 %). LBH-589 induced a significant but weak caspase 3 cleavage in both cell lines (10% and 4% in SW982 and SW1353 cells) whereas PXD101 treatment failed to elicit caspase 3 cleavage. Figure 6B shows representative FACS histograms of untreated cells (black filled) versus SAHA treated cells (striated lines), and LBH-589 cells (white filled). The mean percentages of cleaved caspase 3 are summarized in Table 2. In line, western blot analysis revealed distinct PARP cleavage after treatment with the IC_75_ concentrations of SAHA and LBH-589 in both cell lines (Figure 6C), while the effect of PXD101 was less pronounced.

**Figure 6:** HDACi induce apoptosis in sarcoma cells SW-982 and SW-1353 cells were treated with the IC_50_ of SAHA, LBH-589, and PXD101 and **(A)** caspase 3/7 activity was measured in the period from 3-72 h. Data represent mean ± SEM of at least three experiments performed in quadruplicate (*p < 0.05 compared to controls, asterisks are representative for all three drugs). **(B)** Cleavage of caspase-3 was detected after 48 h by flow cytometry. The y-axis denotes cell counts and the x-axis represents fluorescence intensity of FITC antibody. Black curves represent untreated control cells, striated lines show SAHA treated cells, and white curves are LBH-589 treated cells. **(C)** Cells were incubated for 48 h with HDACi at the indicated concentrations. Total cell lysates were subjected to SDS-PAGE and transferred onto PVDF membranes for subsequent detection with anti-PARP. Lysats of Staurosporin (protein kinase inhibitor) treated Jurkat cells (1 μM for 3 h) were used as positive controls for PARP cleavage. Δ represents fold change of cleaved PARP normalized to controls (mean±SD of n = 3).

**Table 2:** Percentage of cleaved caspase 3 positive sarcoma cells after 48 h exposure to HDAC inhibitors (n = 3; mean ± SD; *p < 0.05, **p < 0.01, ***p < 0.001)

Cell line	Treatment	Time	Cleaved caspase 3 (%)
SW-982	*control*	48 h	*1.41±0.73*
	SAHA	48 h	20.76±4.07**
	LBH-589	48 h	10.53±4.42*
	PXD101	48 h	3.85±1.61
SW-1353	*control*	48 h	*1.73±0.44*
	SAHA	48 h	28.31±13.50**
	LBH-589	48 h	4.72±3.06*
	PXD101	48 h	3.54±0.67

### Synergistic effect on chondrosarcoma cells

To determine whether HDACi improve the anti-proliferative effect of the clinically frequently used chemotherapeutic agent doxorubicin, we used its respective IC_50_ values (SW-982: 0.1 μM; SW-1353: 0.5 μM; evaluated by MTS assay, data not shown) in combination with HDACi and measured the cell viability after 48 h using the MTS assay (Figure 6). Whereas in SW-982 cells no synergistic effect could be observed (Figure 7A), in SW1353 cells the combination of doxorubicin with all three HDACi resulted in a significant reduction of cell growth compared to doxorubicin treatment alone (Figure 7B).

**Figure 7:** Synergistic activity of HDACi in combination with doxorubicin **(A)** SW-982 and **(B)** SW-1353 cells were treated with the IC_50_ concentrations of HDACi, the IC_50_ concentration of doxorubicin (Doxo), and a combination of both agents. Cell viability was determined by MTS assay. Bar graphs represent the percentage of cell growth shown as mean±SD of two independent experiments performed in quadruplicate (one-way ANOVA, followed by Bonferroni's post hoc comparison test).

## DISCUSSION

The rationale for the development of HDACi as anticancer drugs is based on their abilities to inhibit tumor cell growth, induce differentiation, and lower the apoptotic threshold in transformed cells [20–22]. The current study demonstrates that different HDACi inhibit the growth of multidrug resistant sarcoma cell lines via G1 cell cycle arrest and can induce apoptosis. The IC_50_ concentrations are in line with data published for other tumor entities. SAHA and PXD101 have been shown to suppress growth of various tumor cells *in vitro* at low micromolar concentrations [23–25]. LBH-589 produces the same effect at low nanomolar concentrations [26].

Class I HDACs (HDAC1, 2, 3, and 8) are expressed ubiquitously in human tissues and participate in many cellular processes, including proliferation, cell cycle, and apoptosis. In a variety of cancers expression of class I HDACs is elevated compared to the respective tissue of origin [20]. However, the overexpression of HDAC does not necessarily predict a poor outcome and the expression levels of HDAC may not indicate sensitivity to HDAC inhibitors or other anticancer drugs [27]. Further work across tumors, including sarcomas, is required for this to be clinically relevant. In light of multiple published phase 1, 2, and 3 studies in solid tumors, it is surprising that this question has yet to be addressed. Both, synovial sarcoma and chondrosarcoma cells expressed class I HDACs and protein expression levels for HDAC1, 2, 3, and 8 did not change in response to HDACi treatment. Only high concentrations of SAHA affected HDAC8 expression in SW-1353 cells.

The effects of various HDACi on sarcomas have not been sufficiently explored yet. Targeting HDACs in rhabdoid tumors and chondrosarcoma cells was shown to induce cell cycle arrest and apoptosis. In addition, a synergistic interaction of SAHA with established anticancer agents could be demonstrated [28–30]. In synovial sarcoma HDACi induced apoptotic effects were reported through activation of EGR-1 transcription factor [31].

Our study focuses on the influence of HDACi on cell cycle and cell cycle regulatory proteins. Two crucial aspects of cell cycle regulation are the presence of DNA structure checkpoints, which arrest the cell cycle in response to DNA damage or incomplete replication, as well as the presence of a ‘commitment point’. This point is also known as the ‘restriction point’ in human cells and is defined as the point after which a cell is committed to enter and progress through the cell cycle independent from environmental signals. Dynamic changes in gene expression as a function of cell cycle progression are regulated by specific cyclin-dependent kinases (CDK). CDKs form a family of serine/threonine protein kinases that are activated at specific points during the cell cycle [32, 33]. CDK protein levels remain stable during the cell cycle, unlike their activating proteins, the cyclins. Cyclin protein levels rise and fall during the cell cycle and in this way they periodically activate CDK by phosphorylation [34]. Activation of CDK4/6-cyclin D and CDK2-cyclin E complexes are essential for entry into S phase [35]. Unlike the other cyclins, cyclin D is not expressed periodically, but is synthesized as long as growth factor stimulation persists [36]. Our protein analysis data confirmed the cell cycle arrest at G1/S checkpoint observed via FACS analysis. Consistent with the inhibition of G1-to-S phase progression, we found decreased cyclin D1 expression and decreased phosphorylation of CDK4 and CDK2 in synovial sarcoma cells in response to SAHA, LBH-589, and PXD101. The same was found in chondrosarcoma cells after SAHA treatment. In line, decreased cyclin D1 mRNA stability and induction of G0/G1 growth arrest has been reported in colon cancer in response to SAHA treatment [37]. Interestingly, cyclin E levels significantly increased after HDACi treatment in synovial sarcoma cells after SAHA, LBH-589, and PXD101 treatment and in SW-1353 cells in response to SAHA. This is contrary to data published for lung cancer cells treated with SAHA [38]. Mitosis is further regulated by cyclin B in complex with CDK1 [39]. Within this study, expression of cyclin B1 and CDK1 was dormant in SW-982 cells and downregulated in SW-1353 in response to HDACi treatment. Cyclin B1 degradation is a well-known consequence of G1/S phase arrest, whereas CDK1 levels remain constant. However, lysosomal degradation of CDK1 was shown in different low tumorigenic carcinoma cell lines after DNA damage [40] and CDK1 downregulation was reported in ovarian cancer in response to SAHA treatment [41]. The most important mechanism of HDACi mediated G1/S arrest is the increased expression of CDK- inhibitor p21 as observed within our study. Although the expression of p21 is under tight control of its transcriptional regulator p53, HDACi can induce p21 expression in a p53 independent way in several cancer cell lines [42, 43]. In endometrial cancers SAHA was demonstrated to increase p21 expression at simultaneous reduction of p53 and cyclin D level as seen here by SAHA, LBH-589, and PXD101 in synovial sarcoma cells and by SAHA in chondrosarcoma cells [44].

An additional anti-tumor pathway of HDACi is the persistent induction of DNA double strand breaks (DSB) in tumor cells as indicated by enhanced levels of phosphorylated histone variant γH2AX, a biomarker of DSB [45]. And although genotoxic stress such as DNA damage can upregulate p53 leading to subsequent induction of p21, no p53 accumulation was observed.

HDACi have been shown to induce cell death by activating extrinsic and/or intrinsic apoptotic pathways in a number of tumor cells [46]. In order to analyze HDACi-induced apoptosis in sarcoma cells, we performed activation assays of the execution pathway proteins caspase 3 and PARP. The most pronounced pro-apoptotic effects were observed for SAHA and LBH-589 in both, synovial- and chondrosarcoma cells, whereas the effect of PXD101 was less clear.

A further property of HDACi is their proposed ability to enhance the anticancer activity of numerous chemotherapeutic agents. The acetylation of core histones results in an open chromatin configuration that is more accessible to DNA-targeting agents, as well as in shifting the balance of pro- and anti-apoptotic genes towards apoptosis [47, 48]. Thus, the full potential of effective drugs may be best realized by combined chemotherapy. Doxorubicin is one of the most commonly used anticancer drugs for the treatment of sarcoma patients. Morgan & Cranmer demonstrated an *in vitro* synergy between ridaforolimus and SAHA in synovial sarcoma cells [49]. SAHA and PXD101 have anti-proliferative and pro-apoptotic effects in mesenchymal tumors depending on the expression level of HR23b [50].

Although doxorubicin remains the standard-of-care agent for treating STS, its activity can be considered modest at best, resulting in a strong desire to partner doxorubicin with other synergistic cytotoxic and noncytotoxic agents. In the present study, we demonstrated for the first time that SAHA, LBH-589, and PXD101 have synergistic effects with the topoisomerase II inhibitor doxorubicin in SW-1353 chondrosarcoma cells. In contrast, HDACi failed to enhance the cytotoxicity of doxorubicin against synovial sarcoma, pointing to some tumor selectivity [29]. Synergistic or at least additive effects combining HDAC inhibitors and DNA-damaging drugs were shown in a number of cancer types [51]. HDACi mediated sensitization of cancer cells to DNA-damaging agents are explained by their ability to enhance decondensation of chromatin and to abrogate DNA double-strand repair. However, the exact mechanism in sarcoma remains to be clarified.

Taken together, our results demonstrated that SAHA and LBH-589 decreased the viability of human synovial sarcoma and chondrosarcoma cells and arrested the cells in the G1/S phase. Furthermore, both SAHA and LBH-589 increased apoptosis and showed a synergistic effect with doxorubicin in chondrosarcoma cells. In conclusion, our results demonstrate the potential value of vorinostat and panobinostat for the development of novel sarcoma therapeutics.

## MATERIALS AND METHODS

### Cell culture

SW-982 (human synovial sarcoma) and SW-1353 (human chondrosarcoma) cell lines were obtained from Cell Lines Service (CLS; Eppelheim, Germany) in August 2015 and cultured in Dulbecco’s-modified Eagle's medium (DMEM-F12; GIBCO^®^, Invitrogen, Darmstadt, Germany), containing 5% fetal bovine serum (FBS; GIBCO^®^, Invitrogen), 1% L-glutamine, 100 units/ml penicillin, 100 μg/ml streptomycin (all GIBCO^®^, Invitrogen), and 0.25 μg amphotericin B (PAA Laboratory, Pasching, Austria). All cell lines were verified by short tandem repeat analysis using the PowerPlex™ 16 System Kit (Promega, Mannheim, Germany). Cells were incubated at 37°C in a humidified atmosphere of 5% CO_2_ and passaged by trypsinization upon reaching confluence.

### Cell viability assay

5×10^3^ sarcoma cells were seeded into 96-well microtiter plates (Brand, Voerde-Friedrichsfeld, Germany). For the dose-response relationship, cells were exposed to 0-15 μM vorinostat (SAHA), 0-5 μM panobinostat (LBH-589) or 0-5 μM belinostat (PXD101) (all Selleckchem, Houston, TX) for 48 h. To assess synergistic effects of HDACi and the DNA topoisomerase II inhibitor doxorubicin hydrochloride (Sigma Aldrich, Vienna, Austria) combinations of the respective IC_50_ concentrations were used. Cell viability was determined with a luminescent MTS assay (CellTiter 96^®^ AQ_ueous_ Assay; Promega) in accordance with the manufacturers’ instructions using a photometer (Spektramax; BMG Labtech., Offenburg, Germany) at the wavelength of 490 nm. The culture medium was used as a negative control. Results were expressed as the mean from three (dose-response) or two (co-treatment) independent experiments (*n* = 3/2, measured in biological quadruplicates) and error bars represent the SD.

### Cell cycle analysis

After incubation with the respective IC_50_ concentration of HDAC inhibitors for 48 h, cells were harvested by trypsinization and fixed with 70% ice cold ethanol for 10 min at 4°C. After washing, the cell pellet was re-suspended in propidium iodide (PI) staining buffer (50 μl/ml PI, RNAse A; Beckman Coulter, Brea, CA) and incubated for 15 min at 37°C. Cell cycle distribution was analyzed by FACSCalibur (BD Biosciences, San Diego, CA) using ModFit software.

### Western blot analysis

For immunoblotting, whole cell protein extracts were prepared with lysis buffer (50 mM Tris-HCl pH 7.4, 150 mM NaCl, 50 mM NaF, 1 mM EDTA, 10-% NP-40, 1% Triton-X and protease inhibitors), subjected to SDS-PAGE (10 or 12%) and blotted onto PVDF membranes (Roth, Karlsruhe, Germany). Primary antibodies against PARP, CDK4, CDK1, cyclin B1, cyclin E, p21, HDAC1, HDAC2, HDAC3, HDAC8, and β-actin were purchased from Santa Cruz Biotechnology (Santa Cruz, CA, US). Anti-p27^Kip1,^ -cyclin D1, -CDK2, -phosphoCDK2 (Thr160), -phosphoCDK4 (Thr172), and -phosphoH2AX (Ser139) were purchased from Cell Signaling Technology (Danvers, MA, US), and anti-p53 from Dako (Glostrup, Denmark). Blots were developed using corresponding horseradish peroxidase- conjugated secondary antibodies (Dako, Jena, Germany) at room temperature for 1 h and the Amersham™ ECL™ prime western blotting detection reagent (GE Healthcare) in accordance with the manufacturer‘s protocol. Chemiluminescence signals were detected by the ChemiDocTouch Imaging System (BioRad Laboratories Inc., Herkules, CA) and images were processed using ImageLab 5.2 Software (BioRad Laboratories Inc.), normalized to their loading controls and expressed as fold-change (Δ) compared to controls.

### Caspase-Glo^®^ 3/7 assay

For caspase 3/7 activity 10,000 cells/well (100μL) were treated with the respective IC_50_ concentration of HDAC inhibitors for 3-72 h and analyzed for caspase 3/7 activation using the Caspase-Glo^®^ 3/7 Assay (Promega) according to the manufacturer's protocol. Briefly, Caspase-Glo^®^ reagent was added to the sample at a 1:1 volume ratio into each well and incubated at room temperature for 30 min under protection from light. Blank values were subtracted from the experimental values to exclude background luminescence and negative controls were used to determine basal caspase activity. Luminescence of each sample was measured using a Luminometer (LUMIstar; BMG Labtech, Ortenberg, Germany). Results were expressed as the mean from three independent experiments measured in biological quadruplicates with error bars representing the standard deviation.

### Caspase-3 apoptosis assay

After incubation with the respective IC_50_ of HDAC inhibitors for 48 h, cells were harvested by trypsinization, fixed with formaldehyde for 10 min at 37°C (2×10^6^ cells/ml), permeabilized with methanol, and re-suspended in incubation-buffer (FBS:PBS 1:200). Activation of caspase-3, a marker for cells undergoing apoptosis, requires proteolytic processing of its inactive zymogen into activated p17 and p12 fragments. The FITC-conjugated monoclonal cleaved caspase-3 (Asp175) antibody (Cell Signaling Technology, Danvers, MA) detects endogenous levels of the large fragment (17/19 kDa) of activated caspase-3 resulting from cleavage adjacent to aspartic acid175. The antibody does not recognize full length caspase-3 or other cleaved caspases. Cells were analyzed by flow cytometry (FACSCalibur™, BD Biosciences, San Jose, CA) performed with FACSDiva software. Histograms were created using FCS3 express software (De Novo software, Los Angeles, CA). Untreated cells, as well as vehicle controls (DMSO) were used as negative control.

### TP53 Sequencing

Genomic DNA was isolated from SW-982 cell line using the Gentra Puregene Buccal Cell Kit (Qiagen) according to the manufacturer's protocol. PCR of the coding exons of TP53 was performed using a primer set designed with Primer 3 software (http://bioinfo.ut.ee/primer3-0.4.0/; primer sequences available upon request) and the HotStarTaq Master Mix Kit (Qiagen). The subsequently generated sequencing reactions were separated on an ABI 3100 Genetic Analyzer and analyzed by usage of ABI PRISM SeqScape® Software (Applied Biosystems).

### Statistical analysis

Data are expressed as mean±SD or mean±SEM. Student's unpaired *t*-test and one-way ANOVA, followed by Bonferroni's post hoc comparison test, was used for analysis of statistical significance (***p < 0.001; **p < 0.01; *p < 0.05). The significance of dose or time responses was assessed by repeated measurements. Graphic data were prepared with GraphPad Prism5. Dose-response data and IC_50_ values were analyzed using a four-parameter logistic model.
